# Short-time QiBaoMeiRan Formula Treatment Exerts Estrogenic Activities without Side Effects on Reproductive Tissues in Immature Mice

**DOI:** 10.1038/srep17436

**Published:** 2015-12-08

**Authors:** Ying Xu, Xiao-ping Ma, Jin-na An, Zi-jia Zhang, Jie Ding, Ya-kun Qu, Zhen-li Liu, Na Lin

**Affiliations:** 1 Institute of Chinese Materia Medica, China Academy of Chinese Medical Sciences, Dongcheng District Dongzhimen Nanxiao Road 16, Beijing 100700, China; 2 The MOE Key Laboratory for Standardization of Chinese Medicines and The Key Laboratory for Pharmacology of Compound Chinese Medicine of Shanghai, Institute of Chinese Materia Medica, Shanghai University of Traditional Chinese Medicine, Shanghai, China; 3 Institute of Basic Theory, China Academy of Chinese Medical Sciences, Dongcheng District Dongzhimen Nanxiao Road 16, Beijing 100700, China

## Abstract

The Chinese herbal preparation QiBaoMeiRan formula (QBMR) displayed estrogenic effects in ovariectomized rats after long-term administration in a previous study. The uterus and vagina are negatively influenced by estrogens in hormone therapy. While QBMR is known to be a phytoestrogen, its estrogenic effects and safety on reproductive tissues after short-term administration and its mechanism via estrogen receptor (ER) pathway haven’t been studied. Here, we characterized its estrogenic effects using immature mice together with *in vitro* studies for further molecular characterization. Immature mice were treated with QBMR at doses of 1.125, 2.25, and 4.5 g/kg for 7 days. 1.125 and 2.25 g/kg QBMR promoted the growth and development of uterus and vagina, and upregulated ERα and ERβ expression in reproductive tissues. QBMR had a stimulatory effect on proliferating cell nuclear antigen in vagina but not in uterus, and was without any influence on ki-67 antigen in uterus and vagina. QBMR significantly induced luciferase expression from the ERα/β-estrogen response element (ERE) luciferase reporter and upregulated ERα and ERβ expressions in MCF-7 cells, which were significantly inhibited by estrogen antagonist ICI182,780. This study demonstrated QBMR exerts estrogenic effects on reproductive tissues without side effects and through ER-ERE-dependent pathway.

In climacteric and postmenopausal women, low serum levels of 17β-estradiol (E_2_) often result in hot flashes, sweating, anxiety, mood swings, as well as an increased risk for many chronic health problems, such as cardiovascular diseases and osteoporosis. These effects have prompted women to receive hormone replacement therapy (HRT) to prevent these aging-associated symptoms or diseases^1^,^2^. In the uterus, E_2_ stimulates endometrial proliferation without the addition of progestin; this stimulation results in endometrial hyperplasia and may possibly lead to neoplasia^3^. The vagina is another target for E_2_, since its epithelium is induced to undergo proliferation and cornification, which are the desired estrogenic effects because lactobacillus use these cells to produce lactic acid to keep the vaginal milieu acidic and thus prevent ascending infections^4^. The uterus and vagina are known to be negatively influenced by estrogens used in HRT. Estrogens alone stimulate endometrial proliferation and may possibly lead to cancer^5^,^6^,^7^, which has led to a search for HRT alternatives, and plant-derived phytoestrogens have been vigorously promoted. Phytoestrogens are similar both structurally and functionally to mammalian estrogens, but with reportedly lower side effects than synthetic HRT^8^,^9^. Phytoestrogens can bind to estrogen receptors (ERs) and appear to have various estrogenic and antiestrogenic effects; therefore, they have been considered as selective estrogen receptor modulators (SERMs)^10^,^11^. Traditional Chinese medicines (TCM) containing multi-interactive compounds, which have been used for centuries in China to treat perimenopausal syndrome, have attracted the attention of researchers interested in using a TCM formula as a new phytoestrogen resource. QiBaoMeiRan formula (QBMR) is recorded in the Chinese Pharmacopeia of 2010 and includes Polygoni Multiflori Radix, Angelicae Sinensis Radix, Achyranthis Bidentatae Radix, Semen Cuscutae, Fructus Lycii, Poria, and Fructus Psoraleae. In our previous study, QBMR exhibited estrogenic activity, as indicated by its interference with the atrophy of reproductive target tissues, such as the uterus, vagina, and mammary gland, in ovariectomized (OVX) rats. In addition, QBMR relieves the symptoms of hot flushes and body weight gain, which are induced by estrogen decline^12^. The Organization for Economic Co-operation and Development recommends that tests for estrogenic activity be performed both in immature and ovariectomized (OVX) rats/mice^13^. Currently, little is known about the biological effects of QBMR on immature mice after short-term oral administration and whether QBMR, as has been reported for phytoestrogens, causes few side effects or whether they are endocrine disruptors that endanger the uterus or vagina. Furthermore, QBMR induces increased ER expression in reproductive target tissues, providing some molecular evidence for estrogenic activity^12^, however, the molecular characterization of the mechanism of action of QBMR via the estrogen receptor has not been characterized. In the present study, we describe the estrogenic effects of QBMR using an *in vivo* model of immature mice and *in vitro* assays in HEK 293 cells stably transfected with hER α/β-the estrogen response element (ERE) plasmid and the ER antagonist ICI182, 780, as part of an ongoing effort to provide scientific data and further identify the mechanism of QBMR’s estrogenic effects.

## Results

### Uterus

#### QBMR promoted the growth and development of the uterus

To characterize the estrogenic effects of QBMR on reproductive targets, we treated immature mice with QBMR and compared the activity to a synthetic estrogen, estradiol valerate (EV). As expected, EV treatment induced a 2.4-fold increase in uterine weight compared to untreated immature mice (p < 0.001). QBMR (1.125 and 2.25 g/kg) significantly increased uterine weight (p < 0.05 or 0.01) and the dose of 2.25 g/kg resulted a maximum of 1.6-fold increase in uterine weight. Notably, the largest dose of QBMR did not decrease uterine weight compared to controls. Rather, it did not stimulate uterine weight (Fig. 1A).

Figure 1B shows microscopic preparations of representative uteri from one animal per treatment group. Histological analysis of uterus sections revealed that immature mice treated with EV or QBMR (1.125, 2.25 g/kg) substantially altered uterine morphology (Fig. 1Bii–v), as indicated by the thickening of the uterine endometrium, increased number of glands, and more extended glandular cavities compared with untreated controls. QBMR 4.5 g/kg decreased uterine cavity and the gland number compared to untreated mice. The morphological findings in the uteri of all animals were quantified and are presented in Table 1. In untreated controls, the endometrium was composed of single layered columnar epithelial cells, and no mitotic activity was detected in epithelial cells. Animals in the QBMR medium group (Fig. 1Bii-iii) endometrial cells were stimulated but no pathological signs were detected. The stromal cells of endometrial lamina propria were well organized and spindle shaped. Endometrial mitotic activity was found in 1 of 10 mice in the QBMR low dose treatment group, in 5 of 10 animals in QBMR higher group, and none in QBMR 4.5 g/kg group. EV (Fig. 1Bv) induced estrogenic features, causing the endometrial epithelium to become multilayered and hypertrophic and the glands hyperplastic in 8 of 10 animals. Mitotic activity was present in the endometrial cells in most animals at various degrees.

#### QBMR increased ERs subtype expression and exerted no effect on PCNA and K i-67 in uterus

Figure 1C shows representative sections of the expressions of ERα, ERβ, PCNA, and Ki-67 in the uteri from each group and their corresponding quantitative analysis. The number of positive-expressing cells was counted and expressed as a percentage of the total number of cells. Treatment with either EV or QBMR 1.125 and 2.25 g/kg induced a clear up-regulation of ERα and ERβ, and the maximum increases were observed in the higher dose treatment groups (both p < 0.001). Meanwhile, ERβ upregulation was stronger than that of ERα (p < 0.05). ERs in the uterus were expressed in the epithelial cells of the endometrium, interstitial cells, and smooth muscle cells in the QBMR-treated or EV-treated groups. EV significantly stimulated the expression of PCNA and Ki-67 (both p < 0.01), whereas QBMR, at the two doses exhibiting estrogenic activity, there was no significant change apparent in these parameters either in the IHC or the bar graphs, and the highest dose caused a slight decrease in PCNA and Ki-67 expression. PCNA and Ki-67 in the uterus were expressed in the epithelial cells of the endometrium and glands in the QBMR- and EV-treated groups.

Further evidence for the interaction of QBMR with the ERs, PCNA, and Ki-67 were obtained by western blot. As shown in Fig. 1D, similar to the immunostaining results, a dose of 2.25 g/kg significantly upregulated the protein expression of ERα by 2.0-fold (p < 0.001) and ERβ by 2.6-fold, (p < 0.001) compared to a 2.8- and 3.3-fold upregulation of ERα and ERβ induced by EV versus untreated immature mice. In addition, ERβ upregulation by QBMR was more than that of ERα (p < 0.05). Meanwhile, EV significantly stimulated the expression of PCNA (p < 0.05) and Ki-67 (p < 0.05) by 20% and 30% increase, respectively, in the uterus compared to those of untreated immature mice, and QBMR had no significant effect on these parameters in the uterus.

### Vagina

#### QBMR promoted vaginal cornification

The estrus cycle of all mice was monitored by daily inspection of vaginal epithelium cell smears. As shown in Fig. 2A, smears of the vaginal epithelium cells of the untreated immature mice consisted of leukocytes, indicating a diestrus. In contrast, the vaginal cells from the immature mice treated with QBMR at doses of 1.125, 2.25 g/kg or EV became keratinized after about 4 days of treatment, which indicates advanced estrus. Moreover, QBMR treatment prolonged the estrus status of the immature mice, suggesting very potent estrogenic activity. However, in 4.5 g/kg QBMR-treated mice, smears of the vaginal epithelium cells consisted of leukocytes that did not change during the treatment period.

#### QBMR promoted the growth and development of vaginal epithelium thickness

Figure 2B shows microscopic preparations of representative vagina from one animal per treatment group, the morphologic findings in vaginas of all animals were quantified and are presented in Table 2. In untreated control and QBMR 4.5 g/kg group, only three to five cell layers were present, and no cornification was observed in 10 of 10 mice. Compared to untreated immature mice, the EV-treated animals (Fig. 2B v) displayed a typical squamous multilayered epithelium. Approximately 10 ~ 15 cell layers with cornification were observed in all 10 samples. In 1.125 g/kg QBMR-treated animals, epithelium thickness and the number of cell layers were augmented in some areas, and cornification was observed in 8 of 10 rats. An incipient cytoplasmatic vacuolization of epithelial cells was observed in 4 of 10 rats. Treatment with 2.25 g/kg QBMR (Fig. 2B iii) increased epithelial thickness and the number of cell layers (10 layers). Cornification was found in 9 of 10 animals, and no cytoplasmatic vacuolization was noted in all samples. Taken together, these studies provide evidence that QBMR has significant estrogenic potential in the vagina, which is weaker comparable to that of the synthetic estrogen EV.

#### QBMR increased ER subtype and PCNA, and exerted no effect on Ki-67 expression in vagina

Figure 2C shows that treatment with either EV or QBMR at 1.125 or 2.25 g/kg induced clear and comparable up-regulation of ERα and ERβ in the vagina (both p < 0.001). ERs in vagina were expressed in the vaginal epithelium cells of squamous and smooth muscle cells. EV significantly stimulated the expression of PCNA (p < 0.001) and Ki-67 (p < 0.05), 1.125 and 2.25 g/kg QBMR were effective in upregulating the expression of PCNA (p < 0.01), and exerted no effect on K i-67 expression in the vagina, and QBMR 4.5 g/kg did not resulted significant changes in these parameters compared with untreated controls.

The western blot results in Fig. 2D clearly showed that compared to the control group, treatment with QBMR (2.25 g/kg) stimulated levels of ERα and ERβ 1.8- and 2.7-fold, respectively, in the vagina. Similarly, EV induced a 2.1- and 3.3-fold increase in ERα and ERβ in the vagina. Similar to the PCNA- and Ki-67-immunostaining results, EV significantly stimulated PCNA (p < 0.001) and Ki-67 (p < 0.01) expression by 50% and 40% increase in the vagina, respectively, compared to that of untreated immature mice, and the highest dose of QBMR (2.25 g/kg) had a significant effect on protein expression with a 25% increase in PCNA (p < 0.01), and exerted no influence on Ki-67 expression in the vagina.

#### QBMR increased E_2,_ and decreased LH and FSH in serum

Immature mice are expected to have lower levels of serum E_2_, and this is indicated in Fig. 3. Treatment of immature mice with QBMR at any doses or with EV raised levels of circulating E_2_ compared to those of untreated mice (all p < 0.01). QBMR (2.25 g/kg) and EV treatment induced 2.2- and 2.7-fold increases in circulating E_2_, respectively (Fig. 3A). QBMR 1.125 and 2.25 g/kg significantly decreased the levels of serum LH and FSH, and at the higher dose exhibited significantly decreases in LH (37% reduction) and FSH (44% reduction) (Fig. 3B,C), which was a less effect comparable to the decrease induced by EV treatment.

#### QBMR stimulated MCF-7 cell proliferation

To investigate the molecular basis of QBMR activity in more detail, we used MCF-7 human breast cancer cells as a model because they are dependent on estrogen for growth in monolayer culture. An ethanol extract of QBMR, QBMRE, was assessed for its effect on cell proliferation because QBMR powder is not soluble. Because the growth assays were not set up as one single experiment and plating densities varied, comparisons were made by expressing the results as the percentage number of doublings compared to the DMSO as control. Intermediate concentrations of QBMRE and 0.01 μM 17β-estradiol both stimulated proliferation (Fig. 4), demonstrating the estrogenic activity of the QBMR extracts, which were significantly inhibited by the specific ER antagonist ICI 182, 780.

#### QBMR induced both ERα and ERβ transcriptional activity

HEK 293 cells that had been stably transfected with the hERα/β-ERE-luciferase plasmid were used to measure the formation of functional hERα/β-ERE complexes in response to treatment with the QBMR extracts and/or individual compounds. Results are expressed relative to expression in DMSO-treated cells. QBMR increased both ERα and ERβ-ERE luciferase activity in a dose-dependent manner (Fig. 5A). QBMR extract at 0.1 mg/mL induced a 7.26-fold increase in ERα and a 23.4-fold increase in ERβ luciferase activity, which were comparable to the 7.3-fold increase in ERα and 27.5-fold increase in ERβ luciferase activity induced by 17β-estradiol at 0.01 μM. These effects were ablated when treatments were administered in the presence of the specific ER antagonist ICI182, 780, resulting in 84% and 96% inhibition of ERα and ERβ expression in cells treated with 0.1 mg/mL QBMR extract, respectively, which is comparable to that observed with 17β-estradiol treatment. These data indicate that QBMR clearly has estrogenic activity that is mediated through the activation of ERs. Moreover, Fig. 5B showed that QBMRE at any doses significantly increased ERα-ERE-luciferase activity induced by 17 β-estradiol, whereas competitively activated ERβ-ERE-luciferase expression along with 17 β-estradiol. These results shown QBMRE had a dual action on ERα and ERβ but preferentially activated ERβ.

#### QBMR upregulated ER subtype expression in MCF-7 cells

Further evidence for the interaction of the QBMR extract with the ER system was sought by determining the effect of the extract on ER subtype expression in MCF-7 cells by western blotting. The results show that 0.1 mg/mL QBMRE upregulated ERα and ERβ expression by 1.96- and 2.2-fold, respectively. ERα and ERβ expressions were upregulated slightly less by QBMRE than by 17β-estradiol (Fig. 6). The effects of QBMR extract were significantly inhibited by the specific ER antagonist ICI182, 780, with a 47% decrease in ERα and a 29% decrease in ERβ, compared to a 63% decrease in ERα and a 30% decrease in ERβ induced by 17β-estradiol, suggesting that QBMRE mediates estrogenic activity via the ER pathway. Moreover, ERβ upregulation by QBMRE was stronger than that of ERα (p < 0.05).

## Discussion

This study aimed to investigate the estrogenic effects and safety of QBMR on the uterus and vagina in immature mice after short-term administration, and molecular mechanism of its effect via the estrogen receptor pathway. The results show that QBMR promoted the growth and development of the uterus and vagina, upregulated ERα and ERβ expressions in reproductive target tissues, and had a stimulatory effect on PCNA in vagina but not in uterus, and without any effects on ki-67 antigen in reproductive tissues. QBMR was shown to exert its estrogenic activity via the ER-ERE-independent signal transduction pathway.

Previous studies have addressed the effects of QBMR on estrogen target tissues, hot flashes, and weight gain in OVX rats after a relatively long duration of application. Reports about effects after short-term administration, particularly concerning safety, are scarce. Hence, we observed the expression of PCNA and Ki-67 in the uterus and vagina of immature mice treated with QBMR. PCNA is a nuclear protein that is expressed in proliferating cells during the S phase of the cell cycle and is a useful tool in mammary, cervical, and endometrial cancer prognosis research^14^,^15^. Protein of proliferation intensity (Ki-67-antigen) is an excellent marker for determining the growth cell fraction of a given cell population^16^. The number of PCNA- and Ki-67-positive cells in the uterus and vagina significantly increased in the EV-treated group compared to the vehicle-treated group. PCNA and ki-67 analysis also indicates that QBMR has a clear stimulatory effect on the vagina but not on the uterus compared to the control untreated group. The data reveal that estrogenic responses induced by QBMR show tissue variation that may reflect different affinities of PCNA and Ki-67 for QBMR components. Stimulated uterus cell proliferation is a risk factor for the development of cancer^17^, and the PCNA and ki-67 cell proliferation marker results suggest that QBMR treatment for a short time is maybe safer in the uterus than EV treatment. Moreover, ERα is required for the development of cervical and vaginal cancers, long-term use of drugs that consist of more components acting as ERα-selective agonists could increase the risk of carcinogenesis^18^. It has been reported that ERα and ERβ produce opposite effects on human breast cancer cell proliferation and tumor formation^19^. ERα mediates the breast cancer-promoting effects of estrogens, and ERβ mediates its inhibitory effects. The ERα:ERβ ratio changes during the process of tumorigenesis with an increase in ERα and a decrease in ERβ expression. This phenomenon has been observed in relation to breast^20^, colon^21^, and prostate^22^ cancers. We found that QBMR upregulated ERβ expression more significantly than ERα in the uterus (Fig. 1C,D) and vagina of immature mice (Fig. 2C,D), and the same effects on ERs subtype were also found in OVX rats after a long QBMR treatment^12^. These results suggesting that QBMR could induce agonistic or antagonistic effects depending on target organs, such as SERM, and QBMR was safe for reproductive target tissue, maybe owing to a balanced ratio of ERα:ERβ. Mammary gland is one target for estrogen; however, compared to our previous study, we did not observe the effect on mammary gland because of the limited sample number of immature mouse models available.

Doses of QBMR were calculated based on guidelines published by the Center for Drug Evaluation and Research of the U.S. Department of Health and Human Sciences, in which estimates are given for equivalent doses in humans and common laboratory animals. The highest dose selected in the present study was based on a recommended dose of 0.45 g/kg in humans, but the dose dependency of some responses suggests that the range of doses could have been extended to lower doses. Of the three doses of QBMR used, the middle dose, 2.25 g/kg, induced the most profound physiological responses in immature mice. The highest dose of QBMR 4.5 g/kg, only increased serum estradiol and decreased LH and FSH levels, albeit to a lesser extent than the lower dose. These responses were not accompanied by promotions in the development of uterus and vagina tissue and the upregulation of ERs in target tissue. The weaker responses elicited at the highest doses suggest that these doses are on the downward slope of a bell-shaped, or biphasic, dose-response relationship consistent with some phytoestrogens^23^, which also suggest QBMR maybe is safe for reproductive tissues of immature mice in a short treatment because without increasing response accompany with increasing dose. Interestingly, in our previous OVX rat research, the lowest dose of QBMR induced the most profound physiological response in decreasing hot flashes^12^. The data suggest that estrogenic responses induced by QBMR show tissue variation that may reflect different affinities of ERs for QBMR components.

Estrogens are mainly synthesized in the ovary. The increased serum estrogen concentration after treatment with QBMR suggests that the effect of QBMR may be mediated through the hypothalamus-pituitary-ovary axis and stimulate the biosynthesis of estrogen in the ovary. Meanwhile, QBMR could increase the serum estradiol level in OVX rats in our previous study^12^. It is worth mentioning that the stimulation of estrogen synthesis in premature ovarian failure animals when they were administrated by other phytoestrogens^24^. Moreover, the increase in serum estradiol levels cause a decrease in FSH and LH production by inhibiting or negative feedback of GnRH production in the hypothalamus^25^,^26^. Our results suggested QBMR induced higher estrogen release and inhibited the secretion of FSH and LH maybe by negative feedback regulation.

Estrogen mediates its actions by binding to the ER and inducing a major conformational change, causing the estrogen-ER complex to relocate to the nucleus to bind to its cognate DNA response element (ERE) located in the promoter/enhancer regions of target genes, allowing the regulation of gene transcription^27^,^28^. Under physiological conditions, the biological effects of estrogen depend not only on estrogen levels, but also on the distribution and expression levels of the corresponding ERs in the target cell, ERα, and ERβ^29^,^30^,^31^,^32^,^33^,^34^. The MCF-7 cell line expresses ERs and is dependent on estrogen for proliferation in monolayer culture^35^,^36^,^37^. Using an ethanol extract of the complete QBMR formula, we found that QBMRE at the two intermediate doses induced moderate proliferation of MCF-7 cell. At the same concentrations, QBMRE could significantly stimulate the activity of an ERα/β-ERE–luciferase reporter gene in HEK 293 cells. QBMR was more effective at stimulating the ERβ-ERE luciferase reporter than ERα- ERE luciferase reporter. Both QBMRE and agonist activity were strongly inhibited by the ER antagonist ICI182, 780, which suggests that QBMR exhibited estrogenic activities via the ERE pathway by interacting with the estrogen receptor. Similar effects were found on the expression levels of ERs in MCF-7 cells, in which QBMRE induced an upregulation of ERα and ERβ, similar in magnitude to the estrogen agonist 17β-estradiol, and all responses were inhibited by ICI182, 780. ERβ upregulation induced by QBMRE in MCF-7 cell was stronger than that of ERα (Fig. 6), which also corresponds with ERs transcriptional activity detection in HEK 293 cells with stably transfected the hERα/β-ERE-luciferase plasmid (Fig. 5). Based on the increases of ERβ expression by QBMR than that of ERα in the uterus (Fig. 1C,D) and vagina of immature mice (Fig. 2C,D), suggesting that QBMR maybe bind to ERβ with higher selectivity than ERα. Other phytoestrogens have also been reported to have a higher affinity and selectivity for ERβ^38^. Long-term use of those drugs that consist of more components acting as ERα-selective agonists could increase the risk of carcinogenesis^30^, which may explain why phytoestrogen is safer than HRT.

This study provides evidence that QBMR acts as an estrogen agonist. Further studies are in progress in our laboratory to investigate the use of QBMR as an effective dietary supplement to improve the quality of life for menopausal women and to identify the estrogenic compounds in the QBMR.

## Materials and Methods

### *In vivo* studies

#### Animals and experimental design

The experimental protocol was approved by Institute of Chinese Materia Medica, China Academy of Chinese Medical Sciences and all methods were carried out in accordance with the approved guidelines.

Female, 21-day-old, immature mice (12 ± 2 g) were purchased from Experimental Animal Center of Academy of Military Medical Sciences (Certificate No. SCXK [Jun] 2012-0004). The immature mice were randomly assigned to five groups: control group (Con, n = 10), immature mice were oral administrated with 0.154 mg/kg estradiol valerate or intragastrically at a daily dose of 1.125, 2.25, or 4.5 g/kg (QBMR, n = 10 in per group) for 7 days. Dose calculations followed guidelines correlating the dose equivalents between humans and laboratory animals based on ratios of body surface area. Untreated control mice received distilled water only.

#### Herbal preparation

QBMR was prepared as described in the Chinese Pharmacopeia of 2010. Briefly, the seven ingredients, including Polygoni Multiflori Radix (128 g), Angelicae Sinensis Radix (32 g), Achyranthis Bidentatae Radix (32 g), Semen Cuscutae (32 g), Fructus Lycii (32 g), Poria (32 g), and Fructus Psoraleae (16 g), were pulverized to a fine powder, suspended in distilled water to a concentration of 0.45 g/mL, and the contents of the representative chemical compositions were described in our previous report^12^. The sample for cell culture assays was prepared by extracting the powder with eight-fold volume of 70% ethanol (three, times, for 1 h each). The combined extracts (QBMRE) were concentrated *in vacuo* and dissolved in DMSO (1 g/mL). The contents of representative chemical compositions in QBMRE for cell culture were determined by HPLC. The data were obtained using an Agilent 1200 Series HPLC with DAD. A Zobax SB-C18 column (4.6 mm × 250 mm; 5 μm; Agilent Technologies, Santa Clara, CA, USA) was used. The mobile phase consisted of 0.1% formic acid (A) and methanol (B) with a gradient elution flow rate of 1.0 mL/min. The gradient program (A/B, v/v) was as follows: 93:7 (t = 0 min), 42:58 (t = 18 min), 35:65 (t = 18.5 min), 35:65 (t = 30 min), 0:100 (t = 30 min), and 0:100 (t = 50 min). The detection wavelength program was 320 nm (t = 0 ~ 17 min), 316 nm (t = 17.01 ~ 18.30 min), 250 nm (t = 18.31 ~ 21.00 min), 246 nm (t = 21.01 ~ 28 min), and 254 nm (t = 28.01 ~ 40 min). The column temperature was set to 40 °C. The HPLC chromatogram is shown in Fig. 7. The contents of 2,3,5,4′-stilbeneglucoside (0.054%), ferulic acid (0.00036%), β-ecdysone (0.00044%), psoralen (0.0021%), quercetin (0.0021%), isopsoralen (0.0012%), emodin (0.0027%), and physcion (0.0017%) in QBMR ethanol extracts were determined.

#### Analysis of vaginal cornification, target tissue, and serum sex hormones

Vaginal epithelium cell smears were performed for every mouse during the 7-day administration period^12^, and keratinized vaginal cells visualized by microscopy were considered indicative of estrus. All mice were sacrificed by decapitation after 7 days of treatment. Blood was collected from the eyeball and 50μL serum for analysis of estradiol (E_2_), follicle-stimulating hormone (FSH) and luteinizing hormone (LH) levels by enzymelinked immunosorbent assay (ELISA) (Beijing Xinfangcheng Biotechnology, China)^39^. The sensitivities of the three ELISA assays were 1.0 pg/ml, 1.0 mIU/ml and 1.0 ng/ml respectively and not soluble structural analogues with other cross-reaction, and all the intra-assay and inter-assay variation of each hormonal assay were less than 9% and 15%.

The uterus and vagina were removed and weighed. The left horns of the uterus and the upper portion of the vagina were stored at −80 °C for analysis by western blot. The right horns of the uterus and the under portion of vagina were fixed with 4% polyoxymethylene for 24 h. All samples were embedded in paraffin and prepared for cross sections; sections 4-μm thick were cut, mounted, and stained with Hematoxylin & Eosin (HE) for microscopy (Olympus, Tokyo, Japan)^40^.

#### Immunohistochemistry

The immunohistochemistry protocol and semi-quantitative analysis were carried out as described in our previous study^12^. The following antibodies were used^12^,^23^,^39^: rabbit anti-estrogen receptor-α polyclonal antibody (1:20, SC-542, Santa Cruz Biotechnology, Santa Cruz, CA, USA), rabbit anti-estrogen receptor-β polyclonal antibody (1:50, ab3577, Abcam Biotechnology, Cambridge UK), rabbit anti-proliferating cell nuclear antigen (PCNA) polyclonal antibody (1:15, SC-7907, Santa Cruz Biotechnology), and rabbit anti-ki-67 polyclonal antibody (1:200, SC-7907, Santa Cruz Biotechnology) were used. The Image-Pro Plus 6.0 System image analysis system was used for quantitative analysis.

#### Western blot

The western blot protocol and semi quantitative analysis were carried out following the protocol of our previous study^12^. The following antibodies were used^12^,^23^,^39^: rabbit anti-estrogen receptor-α polyclonal antibody (1:200, SC-542, Santa Cruz Biotechnology), rabbit anti-estrogen receptor-β polyclonal antibody (1:1000, ab3577, Abcam Biotechnology), rabbit anti-PCNA polyclonal antibody (1:200, SC-7907, Santa Cruz Biotechnology), rabbit anti-ki-67 polyclonal antibody (1:100, SC-7907, Santa Cruz Biotechnology), and rabbit anti-glyceraldehyde 3-phosphate dehydrogenase (GAPDH) monoclonal antibody (1:1000, SC-7907, Cell Signaling Technology, Danvers, MA, USA). The relative quantity of each antibody was measured by Alpha Ease FC (Fluorchem FC_2_) software. The density ratio of protein to GAPDH was calculated from the band density.

### *In vitro* studies

#### MTT assay of MCF-7 cell proliferation

The MCF-7 cell line was purchased from Xiehe Cell Research Institute of Peking Union Medical College (from the American Type Culture Collection [ATCC]) and maintained in Dulbecco’s modified eagle’s medium (DMEM) and 10% heat-inactivated fetal bovine serum (FBS; v/v). To minimize the effects of endogenous estrogens, cells were primed for at least 2 days in Phenol Red-free medium containing 5% charcoal-stripped FBS, and then seeded (2 × 10^3^ cells/180 μL/well) in 96-well plates. Cells were preincubated overnight in estrogen-depleted medium and test samples of QBMR extract (20 μL at varying concentrations in DMSO), 17β-estradiol, the test samples with ICI182, 780 and 0.1% DMSO solvent blank (the same final concentration of DMSO in QBMR and 17β -estradiol solutions) were added and incubated at 37 °C for 2 days. Proliferation was determined by the MTT 3-(4,5-dimethylthiazol-2-yl)-2,5-diphenyltetrazo- lium bromide assay at 490 nm. Percent growth induction was calculated as a percentage of the average response of the DMSO control samples. Results reported are the mean ± standard deviation of four replicate determinations from a representative assay.

#### Transfection and reporter assay of estrogen receptor-subtype selectivity

HEK 293 cells were stably transfected with human estrogen receptor α/β (hER α/β) and the estrogen response element (ERE) plasmid (kindly provided by Professor Yung-Chi Cheng, Yale University), and the luciferase reporter assay system from Promega (WI, USA) was used to evaluate the formation of functional ER α/β -ERE complexes. The cells were maintained and primed to minimize the effects of endogenous estrogens as described above and then seeded (1 × 10^5^ cells/100 μL/well) in 96-well plates. The test samples with or without ICI182, 780 and 17β-estradiol were added to three replicate wells, as described for the MTT assay of MCF-7 cell proliferation, and was incubated for 24 h. Finally, the growth medium was carefully removed and 50 μL of lysis buffer per well was added, and the plate was rocked for 15 min. Twenty microliters of the detached cell solution was then transferred to a white micro well plate. Luciferase assay reagent (50 μL) was added to each well, and luciferase activity was measured immediately. Activity of the luciferase reporter gene was expressed relative to the DMSO control. Results reported are the mean ± standard deviation of three replicate determinations from a representative assay.

#### Measurement of ERα and ERβ expression

MCF-7 cells were depleted of E_2_, as described above, preincubated overnight in estrogen-depleted medium at a density of 1 × 10^6^ cells per dish, and then treated with QBMR (0.1 mg/mL) or 17β-estradiol (0.01 μM) with or without 0.1 μM ICI182, 780 and 0.1% DMSO treatment as negative control. All cells were incubated for 48 h and were harvested protein. The western blot protocol and semiquantitative analysis were carried out using the following protocol: ERα antibody (1:200, SC-542 Santa Cruz Biotechnology) and ERβ antibody (1:1000, ab3577, Abcam Biotechnology) were used, and GAPDH antibody (1:1000, SC-7907, Cell Signaling Technology) was used as internal control. All experiments were performed in triplicate. Mean normalized protein expression ± S.E. was calculated from independent experiments.

## Statistics Analysis

The SPSS software version 11.0 for Windows (SPSS Inc, Chicago, IL, USA) was used for statistical analysis. All data were expressed as mean ± standard deviation and were analyzed by one-way analysis of variance (ANOVA) followed by least significant difference (LSD) or Dunnett’s T3 test. Differences were considered statistically significant when p was less than 0.05.

## Additional Information

**How to cite this article**: Xu, Y. *et al.* Short-time QiBaoMeiRan Formula Treatment Exerts Estrogenic Activities without Side Effects on Reproductive Tissues in Immature Mice. *Sci. Rep.* **5**, 17436; doi: 10.1038/srep17436 (2015).

## Figures and Tables

**Figure 1:** The effects of QiBaoMeiRan formula (QBMR) on uterus. Data are the mean ± standard deviation (SD) of samples from 10 mice. P values are based on the results of a one-way analysis of variance (ANOVA) comparing the treatment group to untreated immature mice. ***p < 0.001 **p < 0.01 and *p < 0.05, compared to the control group. #p < 0.05, compared with 1.125 g/kg group. (▲) p < 0.05, compared with ERα protein relative increase to Control. (**A**) The weights of uters were measured at the end of the 7-day treatment period. (**B**) The effects of QBMR treatment on the histology of the uterus in immature mice. Representative photomicrographs taken at 200× and 400× magnification. Insets (Fig. 1Bi-iv) show higher magnifications of endometrium (arrowhead). The square in (Fig. 1Bv) indicates the area shown at higher magnification in (Fig. 1Bvi). (**C**) The effects of QBMR treatment on the expression of the estrogen receptor (ER) α, ERβ, proliferating cell nuclear antigen (PCNA) and ki-67 antigen in the uterus. Representative photomicrographs taken at 200× magnification of ERα, ERβ expression in the uterus, 100× magnification of PCNA and ki-67 expression in uterus sections from each treatment group are shown: (i) untreated immature mice, (ii) 1.125 g/kg, (iii) 2.25 gr/kg, (iv) 4.5 g/kg QBMR, and (v) estradiol valerate (EV). (**D**) The effects of QBMR on the protein expression levels of estrogen receptor (ER) α, ERβ, proliferating cell nuclear antigen (PCNA) and ki-67 in the uterus by western blot and the analyses were carried out as described in the Materials and Methods.

**Figure 2:** The effects of QiBaoMeiRan formula (QBMR) on vagina. Data are the mean ± standard deviation (SD) of samples from 10 mice. P values are based on the results of a one-way analysis of variance (ANOVA) comparing the treatment group with untreated immature mice. ***p < 0.001 **p < 0.01 and *p < 0.05, compared to the control group. #p < 0.05, compared to QBMR 1.125 g/kg group. (▲) p < 0.05, compared with ERα protein relative increase to Control. (**A**) The effects of QBMR on the estrus cycle. Vaginal epithelial cell smears were taken at the seventh day from immature untreated mice (i), mice treated with QBMR 1.125 g/kg (ii), mice treated with QBMR 2.25 g/kg(iii), mice treated with QBMR 4.5 g/kg (iv), and mice treated with estradiol valerate (EV) (v). (**B**) The effects of QBMR treatment on vagina histology in immature mice. (**C**) The effects of QBMR treatment on the expression of ERα, ERβ, and PCNA in the vagina. Representative photomicrographs taken at 400× magnification of the uterus, ERα and ERβ expression in the vagina, 100× magnification of PCNA and ki-67 expression in the vagina sections from each treatment group are shown: (i) untreated immature mice, (ii) 1.125 g/kg, (iii) 2.25 g/kg, and (iv) 4.5 g/kg QBMR, and (v) EV. (**D**) The effects of QBMR formula on the protein expression levels of estrogen receptor (ER) α, ERβ, proliferating cell nuclear antigen (PCNA) and ki-67 in the vagina by western blot.

**Figure 3:** The effects of QiBaoMeiRan formula (QBMR) on serum estradiol (E_2_), luteinizing hormone (LH), and follicle-stimulating hormone (FSH) in immature mice. Serum levels of E_2_ (**A**), LH (**B**), and FSH (**C**) were measured at the end of the treatment period. Data are the mean ± standard deviation (SD) of samples from 10 rats. P values are based on the results of a one-way ANOVA comparing the treatment group with untreated immature mice. **p < 0.01, compared to the control group. ^###^p < 0.001, ^#^p < 0.05, compared with QBMR 1.125 g/kg group.

**Figure 4:** Activity of QiBaoMeiRan formula extract (QBMRE) on proliferation of MCF-7 cells. ICI refers to the estrogen antagonist ICI182, 780 and E_2_ to 17β-estradiol. Cell proliferation was carried out as described in the Materials and Methods. Results are expressed relative to the growth of cells treated with 1% dimethylsulfoxide (DMSO). Data are the mean ± standard deviation of quadruplicate analyses, expressed relative to that of treatment with 0.1% DMSO. *p < 0.05, **p < 0.01 compared to DMSO; ^#^p < 0.05, ^##^p < 0.01, compared to QBMRE or 0.01 μM E_2_.

**Figure 5:** Activity of QiBaoMeiRan formula extract (QBMRE) on estrogen receptor (ER) α/β -estrogen response element (ERE) luciferases reporter gene expression. (**A**) The effect of QBMRE on ER α/β - ERE luciferases reporter gene expression in HEK293 cells. (**B**) The effect of the combination of QBMRE and E_2_ on ER α/β - ERE luciferases reporter gene expression in HEK293 cells. Data are the mean ± standard deviation of quadruplicate analyses, expressed relative to that of treatment with 0.1% DMSO. *p < 0.05, **p < 0.01 compared to DMSO; ^#^p < 0.05, ^###^p < 0.001, compared to 0.01 μM E_2_. (▲▲▲) p < 0.001, (▲▲▲) p < 0.01, (▲) p < 0.05, compared with ERα-ERE luciferases reporter gene expression relative increase to Control.

**Figure 6:** Estrogen receptor α (ER α) and ERβ expression in MCF-7 cells. Western blot analysis of ER subtype expression in MCF-7 cells was carried out as described in the Materials and Methods. *p < 0.05, compared to DMSO; ^#^p < 0.05, ^##^p < 0.01, compared to 0.01 μM E_2_; (△) p < 0.05, compared to QBMRE. (▲) p < 0.05, compared with ERα protein relative increase to Control.

**Figure 7:** Chromatograms for standard substances (**A**) and QiBaoMeiRan formula (**B**) 1. Stilbeneglucoside, 2. Ferulic acid, 3. β-Ecdysone, 4. Psoralen, 5. Quercetin, 6. Isopsoralen, 7. Emodin, 8.Physcion.

**Table 1:** Summary of the physiological and pathological findings in the uteri of immature mice after treatment with E_2_ or QiBaoMeiRan formula (QBMR).

Group	Spindle-shaped Lamina propria cells	Endometrial epithelium with mitosis	Hyperplastic/Hypertrophic glands
Control	1/10	0/10	0/10
QBMR1.125 g/kg	6/10	1/10	0/10
QBMR 2.25 g/kg	9/10	5/10	1/10
QBMR 4.5 g/kg	2/10	0/10	0/10
EV0.154 mg/kg	10/10	10/10	8/10

**Table 2:** Effects of treatment with E_2_ or QiBaoMeiRan formula (QBMR) on morphological features of vagina in immature mice.

Group	Cell layers				Keratinization	Vacuolization	
	1–6	>6 to <10	10	>10		Incipient	Clear
Control	7/10	3/10	0/10	0/10	5/10	0/10	0/10
QBMR1.125 g/kg	3/10	7/10	0/10	0/10	8/10	1/10	3/10
QBMR 2.25 g/kg	2/10	8/10	0/10	0/10	9/10	0/10	0/10
QBMR 4.5 g/kg	8/10	2/10	0/10	0/10	3/10	0/10	0/10
EV0.154 mg/kg	0/10	0/10	3/10	7/10	10/10	0/10	0/10
